The article "Effect of Parecoxib Sodium Combined with Dexmedetomidine on Analgesia and Postoperative Pain of Patients Undergoing Hysteromyomectomy" was retracted in 2023. Reasons: signs of a paper mill; compromised peer review; unreliable results or conclusions.

# Effect of Parecoxib Sodium Combined with Dexmedetomidine on Analgesia and Postoperative Pain of Patients Undergoing Hysteromyomectomy

**DOI:** 10.1155/2022/5123933

**Published:** 2022-10-14

**Authors:** Xiaowei Wang, Yongxue Chen, Yonglei Zhao, Zhigang Wang, Lu Zhao, Junde Hou, Fei Liu

**Affiliations:** Department of Anesthesia, Handan Central Hospital, China

## Abstract

**Background:**

Propofol combined with remifentanil is the most common anesthesia method in laparoscopic hysteromyomectomy. However, whether the combination of the two is helpful to patients undergoing hysteromyomectomy still requires unclear.

**Objective:**

To determine the effect of parecoxib sodium combined with dexmedetomidine on analgesia and postoperative pain of patients undergoing hysteromyomectomy.

**Methods:**

Altogether, 72 patients receiving hysteromyomectomy in our hospital from February 2017 to March 2019 were enrolled. Among them, 35 patients treated with parecoxib sodium were assigned to the control group, while the rest 37 patients treated with parecoxib sodium combined with dexmedetomidine were assigned to the research group. The following items of the two groups were evaluated: visual analog scale (VAS) score, mechanical pain threshold (MPT), Riker sedation-agitation scale (RSAS) score, and expression of serum cortisol and melatonin.

**Results:**

At 12 and 24 h after operation, the VAS score of the research group was lower than that of the control group (*P* < 0.05), and at 6, 12, and 24 h after operation, the MPT of the research group was notably higher than that of the control group (*P* < 0.05). In addition, at 10 min after extubation, the research group got notably lower RSAS score than the control group (*P* < 0.05). Before extubation and at 20 min after extubation, the research group showed notably higher melatonin expression and notably lower serum cortisol expression than the control group (both *P* < 0.05).

**Conclusion:**

Parecoxib sodium combined with dexmedetomidine can effectively control the postoperative pain of patients undergoing hysteromyomectomy, reduce the incidence of agitation, and effectively control serum cortisol and melatonin in them.

## 1. Introduction

Hysteromyoma is the most common benign tumors of female genitalia, with a global incidence of about 34.8% [1]. It mostly occurs in middle-aged and elderly people [2]. According to the statistical results obtained by Pritts et al., there were about 1.1 million new patients with hysteromyoma worldwide in 2015 [3]. One study by Carranza-Mamane et al. [4] has pointed out that the incidence of hysteromyoma is increasing annually, and more and more young people suffer from it. It is estimated that over 10 million patients will suffer from hysteromyoma worldwide by 2050 [5]. Hysteromyoma has always been a clinical research hotspot due to its high incidence. The main symptoms of patients with uterine fibroids are increased menstruation, prolonged menstruation, increased vaginal secretions or vaginal discharge, compression symptoms (such as frequent urination, constipation), etc. As hysteromyoma has no obvious characteristics in the early stage, patients with this disease often do not have significant clinical manifestations, which leads them to miss the best treatment opportunity [6]. Therefore, the clinically reported incidence of uterine fibroids is much lower than the actual incidence of uterine fibroids. As the disease progresses, if the disease cannot be controlled in time, it will not only endanger women's physical health and induce the consequences of hysterectomy, but also affect their psychological state along with the disease. The current treatment of uterine fibroids can be roughly divided into: follow-up observation, drug treatment, surgical treatment, minimally noninvasive treatment, minimally noninvasive surgical treatment including high intensity focused ultrasound (HIFU), and uterine artery embolization. Currently, operation is the most effective treatment for hysteromyoma [7]. As laparoscopic technique develops and comes into use, there is an efficient and minimally invasive method for hysteromyoma, and patients suffer significantly less surgical trauma and have higher acceptance toward surgery [8].

Propofol combined with remifentanil is the most common anesthesia method in laparoscopic hysteromyomectomy. Targeted continuous pumping can control the depth of anesthesia, with the advantages of taking effect quickly and contributing to fast recovery [9, 10]. Patients may suffer from different degrees of hyperalgesia during recovery and are likely to have agitation, which will greatly compromise their postoperative recovery, so it is necessary to use analgesic and sedative drugs [11]. According to studies by Hadi et al. and Lenz et al., parecoxib sodium and dexmedetomidine can effectively alleviate patients' hyperalgesia and agitation during recovery [12, 13]. However, whether the combination of the two is helpful to patients undergoing hysteromyomectomy still requires further study.

Therefore, this study explored the effect of parecoxib sodium combined with dexmedetomidine on analgesia and postoperative pain of patients undergoing hysteromyomectomy, with the goal of providing reference for future clinical practice.

## 2. Materials and Methods

### 2.1. Clinical Data

Altogether, 72 patients receiving hysteromyomectomy in our hospital from February 2017 to March 2019 were enrolled. Among them, 35 patients (mean age of 32.5 ± 6.8 years) treated with parecoxib sodium were assigned to the control group, while the rest 37 patients (mean age of 32.7 ± 6.4 years) treated with parecoxib sodium combined with dexmedetomidine were assigned to the research group. This study was carried out with permission from the Ethics Committee of our hospital.

### 2.2. Inclusion and Exclusion Criteria

The inclusion criteria of the study are as follows: patients clinically diagnosed as hysteromyoma based on abdominal ultrasonography, patients whose myoma location and size were determined, patients ≥20 years old, patients with detailed general clinical data, and those who or whose immediate families signed informed consent forms.

The exclusion criteria of the study are as follows: patients with severe comorbid cognitive or mental disorders, patients who dropped out from the study halfway, patients with comorbid malignant tumor, severe organ dysfunction, infectious diseases, coagulation dysfunction or hypertension, patients unable to cooperate with the evaluation of perioperative pain and other indicators, and patients with contraindications to sedative and analgesic drugs including propofol, remifentanil, parecoxib sodium, and dexmedetomidine.

### 2.3. Anesthesia Methods

Before operation, each patient was required to fast for food and liquids and injected with penehyclidine hydrochloride (0.5 mg) and phenobarbital sodium (0.1 g) to promote his/her muscle relaxation and reduce his/her gland secretion. The patient' airway was evaluated to understand if he/she had difficult airway, and his/her vital signs including respiration, heart rate, and blood pressure were monitored. Anesthesia induction: each patient was injected intravenously with propofol (2 m/kg) and midazolam (0.06 mg/kg) and also injected intravenously with 15 *μ*g sufentanil for analgesia. In addition, rocuronium (0.15 mg/kg) was adopted as muscle relaxant for each patient. For patients operated on for a long time, the muscle relaxant was added intermittently during the operation. After anesthesia induction, each patient was given tracheal intubation, and remifentanil and propofol were pumped into the patient through a micro pump. At the end, the patient was injected intramuscularly with atropine and neostigmine, and the inserted trachea was pulled out when the patient was able to breathe spontaneously. For patients in the control group, 40 mg parecoxib sodium (Pfizer Inc., State Food and Drug Administration (SFDA) approval number: J20080045) was injected intravenously before pneumoperitoneum was established. For patients in the research group, 0.5 *μ*g/kg dexmedetomidine (Guorui Pharmaceutical Co., Ltd., Sichuan, SFDA: 20110097) was injected based on treatment for the control group.

### 2.4. Enzyme Linked Immunosorbent Assay (ELISA) Determination

Fasting venous peripheral blood (4 mL) was sampled from each patient before and after treatment and let to stand at room temperature for 30 min, followed by 10-min centrifugation at 3000 rpm/min to obtain the upper serum. The obtained serum was subpackaged by enzyme-free EP tubes. Some samples were adopted for experiment, and the rest were stored at -80°C. ELISA kits were purchased from Beijing North Biotechnology Co., Ltd., and all steps were carried out strictly according to the kit instructions.

### 2.5. Scoring Criteria

The visual analog scale (VAS) was adopted to evaluate the postoperative pain of each patient [14]. The scale has a full score of 10 points, and a higher score indicates more serious pain and worse pain control effect. The Von Frey Kit was adopted to measure the mechanical pain threshold (MPT) of each patient at different time points as follows: the fiber tip of the detection tool was made to vertically contact with the skin 2 cm around the incision, and the fiber tip was bent for 2 s. The fiber size was increased gradually from 0.4 g, and the increase was stopped when the patient felt tingling pain. The final intensity value (Xf) was recorded. MPT = Xf  ×  maximum likelihood estimation value  ×  logarithmic value of intensity distance. In addition, the Riker sedation-agitation scale (RSAS) was adopted to score the agitation of each patient after recovery. The scoring rules were as follows: 1 point if the patient could not be awaken, and he/she only responded slightly to malignant stimulation, or even had no response; 2 points if the patient was in sedation, responding to physical stimulation, but unable to respond and communicate with instructions; 3 points if the patient was in sedation and drowsiness, could be awaken by mild stimulation, could obey simple instructions, and fall asleep quickly; 4 points if the patient was quiet, could be awaken easily, and could obey instructions; 5 points if the patient was restless and anxious and could be made to recover to a quiet state under promotion of medical staff; 6 points if the patient was in a relatively serious agitation and required repeated persuasion and even protective restriction by medical staff; 7 points if the patient was in a threatening agitation, he/she attacked on medical staff, and cooperation with him/her was difficult to achieve. Riker score ≥ 5 points was defined as agitation.

### 2.6. Outcome Measures

Primary outcome measures are as follows: VAS score, MPT, and RSAS score of each patient were evaluated.

Secondary outcome measures are as follows: the expression of serum cortisol and melatonin in each patient was determined.

### 2.7. Statistical Analyses

In this study, the collected data were analyzed statistically using SPSS20.0 (IBM Corp, Armonk, NY, USA) and visualized into required figures using GraphPad 7. Data distribution was analyzed using the Kolmogorov-Smirnov (K-S) test, and data in normal distribution were expressed as the mean ± standard deviation (Mean ± SD). Intergroup comparison was carried out using the independent-samples *t* test and introgroup comparison was carried out using the paired *t* test. Enumeration data were expressed as the rate (%), analyzed using the chi-square test, and expressed as *χ*^2^. *P* < 0.05 indicates a notable difference.

## 3. Results

### 3.1. Clinical Data

There was no remarkable difference between the research group and the control group in clinical data including age, hypertension history, body mass index (BMI), smoking history, drinking history, place of residence, dietary favor, exercise habit, and course of disease, so they were comparable (all *P* > 0.05).  Table 1.

### 3.2. VAS Score

No notable difference was found between the two groups in VAS score at 6 h after operation (*P* > 0.05), while at 12 and 24 h after operation, the VAS score of the research group was greatly lower than that of the control group (*P* < 0.05) as shown in Figure 1.

### 3.3. MPT of Patients

Before anesthesia induction, no notable difference was found between the two groups in MPT (*P* > 0.05), while at 6, 12, and 24 h after operation, the research group showed notably higher MPT than the control group (*P* < 0.05) as shown in Figure 2.

### 3.4. RSAS Score

There was no notable difference in RSAS score between the two groups at extubation (*P* > 0.05), while the score of the research group was notably lower than that of the control group at 10 min after extubation (*P* < 0.05) as shown in Figure 3.

### 3.5. Expression of Melatonin

According to the determination results of melatonin, the two groups were not notably different in the expression before anesthesia induction (*P* > 0.05), while before extubation and at 20 min after extubation, the research group showed notably higher melatonin expression than the control group (*P* < 0.05) as shown in Figure 4.

### 3.6. Expression of Serum Cortisol

According to the determination results of serum cortisol, the two groups were not notably different in the expression of serum cortisol before anesthesia induction (*P* > 0.05), while before extubation and at 20 min after extubation, the research group showed notably lower cortisol expression than the control group (*P* < 0.05) as shown in Figure 5.

## 4. Discussion

Hysteromyoma is the tumor with the highest incidence in female genitalia, and its pathogenesis has always been a hot clinical research topic. However, there is a lack of clear research on the pathogenesis of hysteromyoma at home and abroad. As modern medical technology advances, gene theory has been gradually verified to be closely related to many tumor diseases [15, 16]. The activation of oncogenes and inactivation of tumor suppressor genes and mismatch repair genes are the basis of tumorigenesis and development. The overexpression of some oncogenes is caused by gene amplification. Moreover, oncogenes may gain selective growth advantages and produce resistance to chemotherapy drugs, which are all factors affecting the prognosis of patients with tumor [17, 18].

In this study, we compared VAS score and RSAS score between the two groups, finding that combination of 0.5 *μ*g/kg dexmedetomidine and 40 mg parecoxib sodium can effectively relieve postoperative pain and allergy and reduce postoperative agitation of patients receiving laparoscopic hysteromyomectomy under general anesthesia of propofol and remifentanil. The occurrence of hyperalgesia is related to the increased sensitivity of spinal dorsal horn neurons. After anesthesia and operation, the postsynaptic potential mediated by N-methyl-D-aspartate receptor increases, while the threshold of action potential decreases. Dexmedetomidine exerts antagonistic effect on N-methyl-D-aspartate receptor, thus inhibiting hyperalgesia. Its inhibitory effect on postoperative hyperalgesia in patients receiving general surgery has also been widely recognized [19, 20]. Parecoxib sodium is a novel COX-2 inhibitor which has been put into clinical use in recent years. It metabolizes into valdecoxib after entering blood and exerts the inhibition of COX-2 activity in peripheral and central nervous system [21]. Some studies have shown that patients undergoing laparoscopic hysteromyomectomy have different degrees of pain hypersensitivity, and the auxiliary use of dexmedetomidine before pneumoperitoneum can significantly ameliorate the reduction of MPT. Both dexmedetomidine and parecoxib sodium can strongly relieve postoperative pain hypersensitivity. The combination of them has better inhibitory effect on pain hypersensitivity at 24 h after operation, and the efficacy difference may be related to the mechanism of drug action [22]. We analyzed the expression of serum cortisol and melatonin in the two groups, finding that before anesthesia induction, the two groups were not greatly different in the expression of them, while before extubation and at 20 min after extubation, the research group showed notably higher melatonin expression and notably lower serum cortisol expression than the control group. Postoperative agitation of patients receiving general anesthesia is mainly manifested as excitement and disorientation. Its mechanism is not completely clear at present, and it may be related to surgical trauma, massive blood loss, postoperative pain, and catheter indwelling. Improper handling may bring about serious complications and may be even life-threatening [23]. Agitation after recovery may be linked to the change of nervous system excitability. Melatonin is a crucial hormone regulating the excitability, but surgery, trauma, and other factors may lead to a decrease in melatonin secretion, inhibiting central excitement and inducting agitation during the recovery period [24].

Through the above study, we have preliminarily verified that parecoxib sodium combined with dexmedetomidine can alleviate agitation, hyperalgesia and postoperative pain in patients undergoing hysteromyomectomy. However, the study still has some limitations. The drug dose is relatively single and the sample size is small. Therefore, we hope to include more samples and increase drug dosage in future research to make our study more comprehensive and supplement our research results.

To sum up, parecoxib sodium combined with dexmedetomidine can effectively control the postoperative pain of patients undergoing hysteromyomectomy and reduce their agitation, which provides reference for future clinical practice.

## Figures and Tables

**Figure 1:** VAS scores of patients at different time points. At 12 and 24 h after operation, the VAS score of the research group was greatly lower than that of the control group. Note: ^∗^*P* < 0.05 vs. research group.

**Figure 2:** Comparison of mechanical pain threshold between the two groups. (a) Comparison of mechanical pain threshold between the two groups before anesthesia induction. (b) Comparison of mechanical pain threshold between the two groups at 6 h after operation. (c) Comparison of mechanical pain threshold between the two groups at 12 h after operation. (d) Comparison of mechanical pain threshold between the two groups at 24 h after operation. Note: ^∗^*P* < 0.05 vs. research group.

**Figure 3:** RSAS score of patients. The RSAS score of the research group was notably lower than that of the control group at 10 min after extubation (*P* < 0.05). Note: ^∗^*P* < 0.05 vs. research group.

**Figure 4:** Expression of melatonin. (a) Comparison of melatonin expression between the two groups before anesthesia induction. (b) Comparison of melatonin expression between the two groups before extubation. (c) Comparison of melatonin expression between the two groups at 20 min after extubation. Note: ^∗^*P* < 0.05 vs. research group.

**Figure 5:** Expression of serum cortisol. (a) Comparison of serum cortisol expression between the two groups before anesthesia induction. (b) Comparison of serum cortisol expression between the two groups before extubation. (c) Comparison of serum cortisol expression between the two groups at 20 min after extubation. Note: ^∗^*P* < 0.05 vs. research group.

**Table 1:** Comparison of clinical data between control group and observation group [*n*(%)].

	The research group (*n* = 37)	The control group (*n* = 35)	*χ* ^2^ or *t*	*P* value
Age (*Y*)	32.7 ± 6.4	32.5 ± 6.8	0.055	0.956
Hypertension history			0.172	0.679
Yes	11 (29.73)	12 (34.29)		
No	26 (70.27)	23 (65.71)		
BMI	22.05 ± 1.24	22.02 ± 1.17	0.106	0.916
Smoking history			0.002	0.963
Yes	15 (40.56)	14 (40.00)		
No	22 (59.46)	21 (60.00)		
Drinking history			0.007	0.995
Yes	18 (48.65)	17 (48.57)		
No	19 (51.35)	18 (51.43)		
Place of residence			0.695	0.405
Urban area	23 (62.16)	25 (71.43)		
Rural area	14 (37.84)	10 (28.57)		
Dietary favor			0.008	0.927
Light	12 (32.43)	11 (31.43)		
Spicy	25 (67.57)	24 (68.57)		
Exercise habit			0.188	0.664
Yes	23 (62.16)	20 (57.14)		
No	14 (37.84)	15 (42.86)		
Course of disease (week)	4.74 ± 1.04	4.92 ± 0.86	0.798	0.427

## Data Availability

The datasets used and analyzed during the current study are available from the corresponding author upon reasonable request.

## References

[1] Donnez J., Hudecek R., Donnez O. (2015). Efficacy and safety of repeated use of ulipristal acetate in uterine fibroids. *Fertility and Sterility*.

[2] Stewart E. A. (2015). Uterine fibroids. *New England Journal of Medicine*.

[3] Pritts E. A., Vanness D. J., Berek J. S. (2015). The prevalence of occult leiomyosarcoma at surgery for presumed uterine fibroids: a meta-analysis. *Gynecological Surgery*.

[4] Carranza-Mamane B., Havelock J., Hemmings R. (2015). The management of uterine fibroids in women with otherwise unexplained infertility. *Journal of Obstetrics and Gynaecology Canada*.

[5] Donnez J., Donnez O., Matule D. (2016). Long-term medical management of uterine fibroids with ulipristal acetate. *Fertility and Sterility*.

[6] Pritts E. A., Parker W. H., Brown J., Olive D. L. (2015). Outcome of occult uterine leiomyosarcoma after surgery for presumed uterine fibroids: a systematic review. *Journal of Minimally Invasive Gynecology*.

[7] Osada H. (2018). Uterine adenomyosis and adenomyoma: the surgical approach. *Fertility and Sterility*.

[8] Tanos V., Berry K. E., Frist M., Campo R., DeWilde R. L. (2018). Prevention and management of complications in laparoscopic myomectomy. *BioMed Research International*.

[9] Ren L. Q., Sun X. X., Guan Y. (2018). Effects of sevoflurane or propofol combined with remifentanil anesthesia on clinical efficacy and stress response in pregnant women with pregnancy-induced hypertension. *European Review for Medical and Pharmacological Sciences*.

[10] Lee H. C., Ryu H. G., Chung E. J., Jung C. W. (2018). Prediction of bispectral index during target-controlled infusion of propofol and remifentanil. *Anesthesiology*.

[11] Horng H. C., Wen K. C., Su W. H., Chen C. S., Wang P. H. (2012). Review of myomectomy. *Taiwanese Journal of Obstetrics & Gynecology*.

[12] Hadi S. M., Saleh A. J., Tang Y. Z., Daoud A., Mei X., Ouyang W. (2015). The effect of KETODEX on the incidence and severity of emergence agitation in children undergoing adenotonsillectomy using sevoflurane based-anesthesia. *International Journal of Pediatric Otorhinolaryngology*.

[13] Lenz H., Raeder J., Draegni T., Heyerdahl F., Schmelz M., Stubhaug A. (2011). Effects of COX inhibition on experimental pain and hyperalgesia during and after remifentanil infusion in humans. *Pain*.

[14] Visual Analogue Scale (2019). Measurement properties of visual analogue scale, numeric rating scale, and pain severity subscale of the brief pain inventory in patients with low back pain: a systematic review. *The Journal of Pain*.

[15] Kesharwani P., Iyer A. K. (2015). Recent advances in dendrimer-based nanovectors for tumor-targeted drug and gene delivery. *Drug Discovery Today*.

[16] Mangraviti A., Tzeng S. Y., Kozielski K. L. (2015). Polymeric nanoparticles for nonviral gene therapy extend brain tumor survivalin vivo. *ACS Nano*.

[17] Zhang L., Morgan R. A., Beane J. D. (2015). Tumor-infiltrating lymphocytes genetically engineered with an inducible gene encoding interleukin-12 for the immunotherapy of metastatic melanoma. *Clinical Cancer Research*.

[18] Costa P. M., Cardoso A. L., Custódia C., Cunha P., Pereira de Almeida L., Pedroso de Lima M. C. (2015). miRNA-21 silencing mediated by tumor-targeted nanoparticles combined with sunitinib: a new multimodal gene therapy approach for glioblastoma. *Journal of Controlled Release*.

[19] Chen Y., Yao Y., Wu Y., Dai D., Zhao Q., Qiu L. (2015). Transcuta-neous electric acupointstimulation allevi-ates remifentanil-induced hyperalgesia inpatients undergoing thyroidectomy : a ran-domized con- trolled trial. *International Journal of Clinical and Experimental Medicine*.

[20] Low Y. H., Gan T. J. (2014). NMDA receptor antagonists, gabapentinoids, *α*-2 agonists, and dexamethasone and other non-opioid adjuvants. *Plastic and Reconstructive Surgery*.

[21] Tomczyk K. M., Wilczak M., Rzymski P. (2018). Uterine rupture at 28 weeks of gestation after laparoscopic myomectomy - a case report. *Przeglad Menopauzalny*.

[22] Afonso J., Reis F. (2012). Dexmedetomidina: papel atual em anestesia e cuidados intensivos. *Revista Brasileira de Anestesiologia*.

[23] Luetz A., Heymann A., Radtke F. M. (2010). Different assessment tools for intensive care unit delirium: which score to use?. *Critical Care Medicine*.

[24] Kuriyama A., Urushidani S., Sato M. (2015). Melatonin and postoperative pain: can the heterogeneous be pooled?. *Anaesthesia*.

